The article "The Oxidant-Scavenging Abilities in the Oral Cavity May Be Regulated by a Collaboration among Antioxidants in Saliva, Microorganisms, Blood Cells and Polyphenols: A Chemiluminescence-Based Study" was published in 2013. Journal: PLoS One.

# The Oxidant-Scavenging Abilities in the Oral Cavity May Be Regulated by a Collaboration among Antioxidants in Saliva, Microorganisms, Blood Cells and Polyphenols: A Chemiluminescence-Based Study

**DOI:** 10.1371/journal.pone.0063062

**Published:** 2013-05-02

**Authors:** Isaac Ginsburg, Ron Kohen, Miri Shalish, David Varon, Ella Shai, Erez Koren

**Affiliations:** 1 The Faculty of Dental Medicine, Institute for Dental Sciences, Hebrew University, Hadassah Medical Center, Jerusalem, Israel; 2 Institute for Drug Research, School of Pharmacy, Richard and Jean Zarbin Chair in Medical Studies, Hadassah Faculty of Medicine, Hebrew University, Jerusalem, Israel; 3 Department of Orthodontics, Hebrew University-Hadassah School of Dental Medicine, Jerusalem, Israel; 4 Coagulation Unit - Hadassah Medical Center, Jerusalem, Israel; University of Toronto, Canada

## Abstract

Saliva has become a central research issue in oral physiology and pathology. Over the evolution, the oral cavity has evolved the antioxidants uric acid, ascorbate reduced glutathione, plasma-derived albumin and antioxidants polyphenols from nutrients that are delivered to the oral cavity. However, blood cells extravasated from injured capillaries in gingival pathologies, or following tooth brushing and use of tooth picks, may attenuate the toxic activities of H_2_O_2_ generated by oral streptococci and by oxidants generated by activated phagocytes. Employing a highly sensitive luminol-dependent chemiluminescence, the DPPH radical and XTT assays to quantify oxidant-scavenging abilities (OSA), we show that saliva can strongly decompose both oxygen and nitrogen species. However, lipophilic antioxidant polyphenols in plants**,** which are poorly soluble in water and therefore not fully available as effective antioxidants, can nevertheless be solubilized either by small amounts of ethanol, whole saliva or also by salivary albumin and mucin. Plant-derived polyphenols can also act in collaboration with whole saliva, human red blood cells, platelets, and also with catalase-positive microorganisms to decompose reactive oxygen species (ROS). Furthermore, polyphenols from nutrient can avidly adhere to mucosal surfaces, are retained there for long periods and may function as a “slow- release devises” capable of affecting the redox status in the oral cavity. The OSA of saliva is due to the sum result of low molecular weight antioxidants, albumin, polyphenols from nutrients, blood elements and microbial antioxidants. Taken together, saliva and its antioxidants are considered regulators of the redox status in the oral cavity under physiological and pathological conditions.

## Introduction

Whole saliva is composed of more than 98% water, a variety of electrolytes, over a thousand different proteins, including the major glycoprotein mucin, plasma-derived-albumin, immunoglobulins, hormones, nucleic acids, digestive enzymes such as alpha-amylase, lysozyme and the nitrogenous products urea and ammonia. Saliva is particularly involved in lubrication, buffering action, maintenance of tooth integrity, physicochemical defense, antimicrobial defense and wound healing, taste and early digestion. It is also important in biofilm formation on tooth surfaces, crystal growth homeostasis, bacterial adhesion, may assist as an important source for genetic and forensic profiles and maintains mucosal integrity of the oral and upper gastrointestinal mucosal surfaces [1].

The article "The Oxidant-Scavenging Abilities in the Oral Cavity May Be Regulated by a Collaboration among Antioxidants in Saliva, Microorganisms, Blood Cells and Polyphenols: A Chemiluminescence-Based Study" was published in 2013. Journal: PLoS One.

Being a portal of entry for nutrients, xenobiotics and colonizing microorganisms, normal saliva is always exposed to a variety of oxidants which might alter the redox status and the integrity of oral structures [1]–[6]. To counteract the toxic effects of oxidants, saliva has evolved a series of low molecular weight antioxidants (LMWA) (e.g. uric acid, ascorbate, reduced glutathione and alpha tocopherol) and antioxidant albumin from plasma is delivered to saliva via the crevicular fluid [7]–[10]. Additional sources of antioxidants in the oral cavity are catalase-positive commensal and fresh blood extravasated from injured capillaries.

Red blood cells have been proposed to act not only as carriers of oxygen and removers of CO_2_ but, also as “sinks” for reactive oxygen species (ROS) and as protectors of other cells against oxidative stresses [11]–[13]. Also, in cases of more massive hemorrhages characteristics of gingival pathologies, exacerbation of tissue damage may occur due to toxic iron-catalyzed hydroxyl radical [3]. Thus, presence of blood in the oral cavity may have a “double-edged sword” effect. We have recently shown [14]–[16] that a variety of microbial species and red blood cells have the capacity to bind to their surfaces a large variety of antioxidant polyphenols from nutrients endowing upon the cells a marked enhancement of oxidant-scavenging abilities (OSA). Red blood cells coated by polyphenols, were also shown to act in concert with salivary low molecular weight antioxidants (LMWA) to enhance the scavenging of ROS, which was further markedly increased either by albumin or mucin both acting as solubilizers of polyphenols making them more effective antioxidants [16], [17]. Also, “sticky” polyphenols in a variety of common beverages were able to avidly bind to oral surfaces and to persist there for long periods despite a constant salivary flow [16]. This phenomenon might explain the potential protective role played by nutritional polyphenols against oxidative stresses in the oral cavity.

The article "The Oxidant-Scavenging Abilities in the Oral Cavity May Be Regulated by a Collaboration among Antioxidants in Saliva, Microorganisms, Blood Cells and Polyphenols: A Chemiluminescence-Based Study" was published in 2013. Journal: PLoS One.

Taken together, we argue that under physiological and especially in pathological conditions, multiple interactions might occur among orally-induced oxidants, salivary antioxidants, antioxidant polyphenols from nutrients, the antioxidants associated with the microbial flora and with blood cells. Such complex interrelationships might affect the integrity of oral tissues especially under inflammatory stresses.

The present study employed mainly a highly-sensitive luminol-dependent chemiluminescence assay, capable of quantifying antioxidants in saliva, whole blood as well as in polyphenolic substances. We also describe the oxidant-scavenging abilities in the oral cavity using additional methodologies such as the DPPH**,** the Folin-Ciocalteu’s reagent and a novel tetrazolium salt assay to quantify polyphenols. We hypothesize that combinations and permutations among a variety of polyphenols, antioxidants present in saliva, blood cells, and in microorganisms may regulate the redox status in the oral cavity under normal and pathological conditions.

## Materials and Methods

### Biochemicals and Plant-derived Agents

Unless otherwise indicated, all the reagents employed were purchased from Sigma-Aldrich (St. Louis, MO, USA). The polyphenols quercetin, catechin, Epigallocatechin gallate (EGCG), gallic acid, caffeic acid, rutin, curcumin, resveratrol, the free radical DPPH (2,2-Diphenyl-1-picrylhydrazyl) were all prepared in absolute ethanol at 100 mM. Tannic acid, gastric mucin, bovine and human albumin, lipopolysaccharide (LPS) from *Escherichia Coli (E. Coli)*, sodium selenite, CoCl_2_, reagent H_2_O_2_ and sodium azide (a catalase inhibitor) were prepared in 0.9% sodium chloride solution (saline). Red wine, green and black tea, roasted coffee, cacao, cinnamon, pomegranate and cranberry drinks were purchased from commercial sources. The Tibetan traditional plant mixture Padma 28 [18] and the Ayurvedic plant preparation Padma hepaten [19] were kindly provided by Padma AG, Shwertzenbach, Switzerland**.** One hundred mg/mL portions of the various herbs were brought to a boiling point and the insoluble fractions were removed by centrifugation. Bradford (Bio-Rad) reagent was used to quantify proteins in saliva using bovine serum albumin (BSA) as a standard and was read at 595 nm [20]. Hank’s balanced salt solution (HBSS) was purchased from Beit-Haemek Industries, Israel.

### Un-stimulated Saliva

Ethics Statement: Ethical and saliva sampling procedures were approved by the Hadassah Medical Center Ethics Committee for Human Subject Research, and a written informed consent was obtained from all participants after an explanation of the study was provided (approval ID 0313-11-HMO). Fasting un-stimulated whole saliva was collected from healthy laboratory personnel ages 23–30 by the spitting method [21], kept on crushed ice and used on the same day. The saliva was expectorated into a small 50 mL sterile plastic vial periodically over 5 min. Saliva was also subjected to centrifugation for 10 minutes at relative centrifugal force (RCF) of 13,000 g in an Eppendorf centrifuge and both the supernatant fluids and the re-suspended precipitates were kept on ice. In some experiments, whole saliva was also dialyzed for 12 hours against saline at 4°C in dialysis tubing bags with a cutoff point of 6 kD. All saliva samples were tested for their OSA employing several analytical assays (see below).

The article "The Oxidant-Scavenging Abilities in the Oral Cavity May Be Regulated by a Collaboration among Antioxidants in Saliva, Microorganisms, Blood Cells and Polyphenols: A Chemiluminescence-Based Study" was published in 2013. Journal: PLoS One.

### Microorganisms

A clinical strain of *Candida Albicans* ***(C. albicans)*** was obtained from the Department of Microbiology, Hadassah Hospital, Jerusalem, Israel. It was grown for 15 hrs. at 30°C on brain heart infusion agar plates. The colonies were scraped off and washed in 0.9% sodium chloride solution. The O.D at 540 nm of the suspensions was adjusted to 20.0 (approximately 10^9^ cells/mL) and used as “carriers” for polyphenols (see **Results** section).

### Red Blood Cells and Platelets

Human heparinized blood and platelets were obtained by consent from the Blood Bank of Hadassah Hospital, Jerusalem, Israel. The cells were washed three times in normal saline, re-suspended in HBSS and used on the same day.

### Preparation of Complexes among Blood Cells, Saliva, Microorgnisms, *Candida* and Polyphenols

Red blood cells (1×107) and *Candida Albicans* (1×108) were incubated for 5 minutes at room temperature with various amounts of polyphenols or of plant extracts (100–200 µM Gallic acid equivalents as quantified by the Folin-Ciocalteu’s reagent). The complexes formed were washed three times in saline and re-suspended in a final volume of 1 mL HBSS. The presence polyphenols bound to cells and the OSA of such complexes were assayed by the luminescence and by the Folin reagent methods respectively (see below).

### Quantification of Polyphenols by the Folin-Ciocalteu’s Reagent

The Folin-Ciocalteu’s reagent is a mixture of phosphomolybdate and phosphotungstate used for the colorimetric assay of phenolics and polyphenolic agents [22]. To 800 µL normal saline were added either washed erythrocytes (1×107) and platelets suspensions (1×107), a variety of microorganisms and also complexes formed among cells, saliva and polyphenols (see above). This was followed by the addition of 50 µL of Folin reagent (Sigma). One minute later, 150 µL of a 25% solution of sodium carbonate were added. This was followed by centrifugation of the reaction mixtures at a low speed (RCF = 250×g) for 3 min and reading the O.D of the supernatant fluids at 760 nm. A standard graph was prepared with gallic acid and the results were expressed as gallic acid equivalents (GAE).

The article "The Oxidant-Scavenging Abilities in the Oral Cavity May Be Regulated by a Collaboration among Antioxidants in Saliva, Microorganisms, Blood Cells and Polyphenols: A Chemiluminescence-Based Study" was published in 2013. Journal: PLoS One.

### Quantification of OSA by Luminol-dependent Chemiluminescence (LDCL) Assays

Two Luminol-dependent chemiluminescence-inducing cocktails [23] were employed to quantify the OSA of un-stimulated saliva, reagent polyphenols, extracts from beverages and plants, whole human blood, washed suspensions of red blood cells (RBC), platelets, a variety of microbial species as well as of complexes made between polyphenols and cells:

- The “H_2_O_2_ cocktail”: is comprised of combinations among 800 µL of Hanks balanced salt solution (HBSS) pH 7.4, luminol (10 µM), H_2_O_2_ (1 mM), sodium selenite (IV) (2 mM) and CoCl_2_ (10 µM). This cocktail generates a constant wave of light due to peroxide and hydroxyl radical [23].
- The “SIN-1 cocktail”: is comprised of combinations among 800 µL of HBSS, luminol (10 µM), morpholino syndononimine (SIN-1) (10 µM), Sodium selenite (1 mM), and CoCl_2_. This cocktail generates a constant flux of light due to the generation of peroxynitrite resulting from the interaction of nitric oxide (NO) and superoxide (See [23]). The degree of light quenching by the various agents indicates their OSA.

### Quantification of OSA by the DPPH Radical Assay

The DPPH radical assay [24], [25] measures hydrogen atom (or one electron) donating activity and hence provides an evaluation of antioxidant activity due to the free radical scavenging, 2,2-Diphenyl-lpicrylhydrazyl radical (DPPH). When reduced, this purple stable free radical, changes its color to a yellow diphenylpicryl hydrazine. In a slightly modified spectrophotometric assay, various agents to be tested (polyphenols, blood cells, saliva, microorganisms) were mixed with 20 µL of a DPPH solution (stock solution of 10 mM in absolute methanol). One minute later, 800 µL of methanol were added. The reaction mixtures were centrifuged at a low speed (RCF = 250×g) for 2 minutes and the change in absorption at 517 nm was determined. Under these conditions red blood cells and platelets (1×107 cells) underwent a prompt fixation but were not hemolyzed. This test can detect reducing agents of a still undefined nature associated with the surfaces of the cells and also of polyphenols bound to cell surfaces.

### Quantification of Antioxidant Capacities by a Tetrazolium Salt Assay

This method is based on the ability of antioxidants to inhibit the reduction of the tetrazolium salt XTT (2,3-Bis-(2-Methoxy-4-Nitro-5-Sulfophenyl)-2*H*-Tetrazolium-5-Carboxanilide) to a pink formazan product, which is read at 450 nm [19]. XTT reduction was induced by a “cocktail” comprised of sodium selenite (2 mM), CoCl_2_ (10 µM) and hydrogen peroxide (1 mM). Briefly, to 800 µL of saline were added XTT (100 µM), various amounts of polyphenols or of un-stimulated saliva. This was followed by the addition of the activating “cocktail” (luminol, selenium, cobalt and H_2_O_2_, see above). The reaction mixtures were kept at room temperature for 10 min, centrifuged and the optical density was measures at 450 nm.

The article "The Oxidant-Scavenging Abilities in the Oral Cavity May Be Regulated by a Collaboration among Antioxidants in Saliva, Microorganisms, Blood Cells and Polyphenols: A Chemiluminescence-Based Study" was published in 2013. Journal: PLoS One.

### Statistical Analysis

Statistical analysis was performed using GraphPad Prism 5 (GraphPad Software, San Diego, CA). The results are presented as mean ± SD. One-way analysis of variance (ANOVA) was applied with the level of significance set at P*<0.05.

## Results

### Levels of Antioxidant Activities in Un-stimulated Saliva

To quantify the OSA of whole un-stimulated saliva, we first employed two highly-sensitive luminol-dependent chemiluminescence assays [23].

**Figures 1a and 1b** show that whole un-stimulated saliva dose-dependently quenched luminescence-induced by oxygen and nitrogen species and that the ID_50_ for the H_2_O_2_ cocktail and SIN-1 cocktail is approximately ∼35 µl and 25 µl saliva respectively. Figures 2a and 2b show that the OSA of saliva can also be assayed, dose-dependently by the XTT and the DPPH radical assays, respectively (see **Materials and Methods**).

**Figure 1:** **a.** Luminol-dependent chemiluminescence patterns of increasing amounts of un-stimulated fasting saliva. Various amounts saliva were added to test tubes containing 800 µL of Hanks balanced salt solution (HBSS). Luminescence was induced by a cocktail comprised of luminol (10 µM), sodium selenite (1 mM), H_2_O_2_ (1 mM) and CoCl_2_ (10 µM). Note the dose-dependent luminescence quenching patterns indicating the ability of salivary oxidants to decompose H_2_O_2_ and hydroxyl radical generated by the cocktail. (n = 10(. **b**. Luminol-dependent chemiluminescence patterns of increasing amounts of saliva tested with the SIN-1 cocktail which generates a constant flux of light due the formation of NO, superoxide and peroxynitrite. Luminescence was induced by a cocktail comprised of luminol (10 µM), sodium selenite, CoCl_2_ (10 µM) and SIN-1 (Morpholino syndonimine (10 µM). Note the dose-dependent inhibition of the generation of light. (n = 5).

**Figure 2:** **a.** OSA of saliva assayed by the XTT reduction method. Increasing amounts of whole saliva in 800 µL HBSS were mixed with XTT (100 µM), followed by the addition of selenite (2 mM), H_2_O_2_ (1 mM) and cobalt (10 µM) (See Materials and Methods). The O.D was read at 450 nm after 10 min incubation at room temperature. (n = 3). **b**. OSA of saliva assayed by the DPPH radical assay. Increasing amounts of whole saliva were added to test tubes containing 20 µL of DPPH (200 µM final concentration.). One minute later, 800 µL of absolute methanol was added and the O.D. of the supernatant was measured at 517 nm. (n = 3)

It was also found (not shown) that while 98% of the OSA of saliva were localized in the supernatant fluid obtained following centrifugation for 5 minutes at relative centrifugal force (RCF) of 13000 g, the “heavy viscous” precipitates, which always contained scattered epithelial cells many of which seeded with micrococci and also leukocytes, had practically no OSA. Furthermore, neither heating saliva to 100°C for 10 seconds, nor freezing at −80°C, affected its OSA. To confirm that salivary antioxidants are mainly associated with low molecular weight agents (urate, ascorbate, GSH) we also subjected saliva to an overnight dialysis against normal saline in casings with a cutoff point of 6 kD. It was found that dialysis of saliva eliminated about 95% of its OSA, confirming that LMWA are mainly involved as antioxidants [1], [7]–[10].

The article "The Oxidant-Scavenging Abilities in the Oral Cavity May Be Regulated by a Collaboration among Antioxidants in Saliva, Microorganisms, Blood Cells and Polyphenols: A Chemiluminescence-Based Study" was published in 2013. Journal: PLoS One.

### Saliva and Ethanol Contribute to the Availability of Polyphenols as Antioxidants

**Figure 3** shows that employing the H_2_O_2_-based luminescence assay tested in aqueous HBSS, non-inhibitory amounts of ethanol nevertheless dose-dependently enhanced OSA of saliva. This might explain the role of ethanol as a solubilizer of red wine polyphenols making them more available as antioxidants [26].

**Figure 3:** Effect of ethanol on salivary antioxidants. Saliva (30 µL) was mixed with increasing amounts of absolute ethanol and the LDCL was measured for 250 seconds. Note: the marked enhancement of luminescence quenching by non-inhibiting amounts of ethanol suggesting that “solubilization” of salivary antioxidants made them more available as antioxidants. (n = 5).

### OSA of Combinations between Saliva and Fruit Beverages

The finding presented in **Figure 3** also led to examine the OSA initiated when a variety of aqueous fruit beverages and reagent polyphenols were combined with saliva. **Figure 4** shows that while using HBSS as a supporting medium, practically all of the “allegedly-soluble” beverages and polyphenols tested showed only a low OSA, a very marked increase in OSA of all agents tested was induced by mixing them with non-inhibitory amounts of fresh saliva. To learn more about the nature of the solubilization of polyphenols by saliva [16] we also tested combinations between polyphenols and the glycoprotein mucin present in high amounts in normal saliva. **Figure 5** shows that mucin very significantly increased the OSA of the polyphenol EGCG. Similar results were also obtained with albumin, a protein considered a “universal carrier” of drugs and metabolites [27], [28] as well as when these proteins were interacted with additional reagent polyphenols (not shown). Our results suggest that both proteins could replace whole saliva as “solubilizers” of polyphenols.

The article "The Oxidant-Scavenging Abilities in the Oral Cavity May Be Regulated by a Collaboration among Antioxidants in Saliva, Microorganisms, Blood Cells and Polyphenols: A Chemiluminescence-Based Study" was published in 2013. Journal: PLoS One.

**Figure 4:** LDCL patterns induced by combinations among saliva (30 µL), a variety of fruit beverages and plant extracts and a polyphenols. All agents fruit beverages were brought to the same gallic acid equivalent (GAE) of 10 µM. P28 is an aqueous extracts from Padma 28 (see Materials and Methods), Hepaten is an aqueous extract from the Ayurvedian traditional plant mixture Padma Hepaten. Hot extracts from Black tea and from double espresso were freshly prepared. Cabernet wine and catechin were dissolved in ethanol. Note that in all cases, low-inhibitory amounts of the various agents acted in a distinct synergistic manner to enhance the antioxidant capacity of 50 µL of saliva. (n = 5).

**Figure 5:** Effect of increasing amounts of gastric mucin on luminol-dependent chemiluminescence (LDCL) quenching by the polyphenol epigallocatechin-3-gallate (EGCG) (17.5 uM). Note that non-inhibitory amounts of mucin dose-dependently increase the antioxidative activity of the tea polyphenol EGCG, presumably by increasing its solubility in aqueous solution. (n = 4).

### Effect of Dialysis on Salivary Antioxidant Activities

Since saliva dialyzed overnight against saline in a dialysis casings with a cut-off of 6 kD to remove LMWA (uric acid, ascorbate and glutathione) lost most of its OSA, we tested whether the high-molecular-weight agents retained in the dialysis bags, which presumably contained high molecular weight mucin, albumin and additional proteins, could still act in concert (synergy) either with added reagent polyphenols or with beverages such as coffee extract, to decompose ROS. **Figure 6** shows that while neither saliva, dialyzed saliva nor extracts from black coffee at the amounts tested, had any appreciable OSA, both whole saliva and dialyzed saliva acted in synergy with a coffee extract to decompose ROS. It suggested, therefore, that salivary high molecular weight agents have the capacity to increase the availability of polyphenols as effective scavengers of ROS.

**Figure 6:** Effect of saliva and of dialyzed saliva on the OSA of coffee extract. Saliva was dialyzed for 15 hours against saline and then tested for its capacity to modify LDCL. Note that while neither saliva, dialyzed saliva (D) nor a coffee extract at 5 µM GAE had any LDCL-quenching abilities, combinations either of saliva and coffee and dialyzed saliva and coffee very markedly quenched luminescence. Data were analyzed by one–way ANOVA and differences were considered significant when P* <0.05, (n = 3).

The article "The Oxidant-Scavenging Abilities in the Oral Cavity May Be Regulated by a Collaboration among Antioxidants in Saliva, Microorganisms, Blood Cells and Polyphenols: A Chemiluminescence-Based Study" was published in 2013. Journal: PLoS One.

### Binding of Salivary Antioxidants to Red Blood Cells

Employing the H_2_O_2_ luminescence assay, **Figure 7** shows a dose-dependent increase in luminescence quenching induced by RBC (5×106) pre-coated by increasing amounts of saliva (50–400 µL) possessing Folin-positive agents at 20–100 µM of gallic acid equivalent (GAE). Similar results (not shown) were also obtained when a variety of washed microbial suspensions were incubated with polyphenols-containing saliva. This suggests the ability of RBC to bind salivary polyphenol antioxidants, which can markedly further increased by consumption of nutrients.

**Figure 7:** Binding of salivary antioxidants by washed RBC. Washed human RBCs (1×107 cells) were added to test tubes containing 800 µL HBSS. This was followed by the addition of saliva. 3 minute later the cells were washed in saline and then tested for their OSA. Note the dose dependent increase in luminescence quenching. (n = 3).

### The OSA of Combinations among Saliva, RBC and Polyphenols

**Figure 8** shows that saliva with low OSA activity nevertheless acted in a synergistic manner with the polyphenol quercetin and with whole blood to decompose ROS. It was also found that sodium azide, a potent inhibitor of heme proteins, totally abolished the stimulatory effect of whole blood (not shown). It is also of interest that similar collaborative responses were also induced when saliva was mixed with washed suspensions of catalase-positive *E. Coli*, *Staph. aureus*, *Pseudomonas Aeuroginosa* (not shown). Since blood pre-treated with sodium azide, an inhibitor of heme proteins, failed to act in concert either with saliva or with mucin to decompose ROS, it was assumed that RBC did not simply act as “solubilizers” of polyphenols but rather as donors of intracellular antioxidants. This also implied that even minor hemorrhages in the oral cavity might contribute potent antioxidants which can act in concert with salivary antioxidants, polyphenols and also with microbial antioxidants (see below and the **Discussion** section) to decompose ROS and thus to improve the antioxidant status in the oral cavity [11]–[13], [29].

**Figure 8:** The combined OSA of saliva, whole blood and Quercetin. Saliva (20 µL) was mixed either with RBC (5×106), quercetin at 10 µM or with combinations among all 3 agents. Note that while neither saliva at very low OSA nor quercetin had any substantial luminescence-quenching abilities, RBC induced a typical bell-shaped pattern of luminescence quenching [15]. However, combinations of RBC and quercetin enhanced luminescence quenching which was nearly maximal when all 3 agents were mixed together. The data imply that RBCs act as potent amplifiers of luminescence quenching a very useful method to detect small amounts of polyphenols. (n = 3).

The article "The Oxidant-Scavenging Abilities in the Oral Cavity May Be Regulated by a Collaboration among Antioxidants in Saliva, Microorganisms, Blood Cells and Polyphenols: A Chemiluminescence-Based Study" was published in 2013. Journal: PLoS One.

### A Long Retention of Antioxidant Polyphenols in Saliva after a Short Exposure of the Oral Cavity to Polyphenol-rich Beverages

Since polyphenols, including tannic acid, are considered “sticky” agents with a capacity to avidly bind to surfaces of microorganisms and of blood cells and to enhance their OSA [13]–[16], it was reasonable to assume that polyphenols in fruit beverages might also avidly bind to the huge surfaces of the oral cavity [16]. These include the tongue, the palate, the gingival epithelium, the teeth and also to the microbial flora. We therefore questioned how long after the exposure of the oral cavity for very short periods to a variety of polyphenols-rich fruit beverages, saliva might still retain enhanced OSA?. To explore this issue, 5 mL amounts of aqueous double-strength espresso, roasted black coffee, black or green tea, cacao, red wine and aqueous extracts from cinnamon all normalized to 50–100 mM GAE, were held in the mouth for 30 seconds and then swallowed. Also, 10 gr. of dark chocolate (60% cacao) was chewed for 30 seconds and then also swallowed. Saliva was then collected at various time intervals thereafter and the levels of OSA were evaluated by the luminescence and by the DPPH assays. In parallel, the polyphenols levels in saliva were also quantified by the Folin reagent. Tested by luminescence, **Figure 9** shows a relatively long persistence of antioxidants activities in saliva following exposure of the oral cavity to a double espresso coffee drink and samples collected even after 120 minutes still contained a higher level of OSA. This suggested that “sticky polyphenol agents”, acted as a “slow release” devises and this, despite a constant salivary flow.

**Figure 9:** A prolonged retention in the oral cavity of antioxidant agents in an espresso drink. 5 mL of an espresso drink containing approximately 45 mM of polyphenols (tested by the Folin reagent) was held in the mouth for 30 seconds and hen swallowed. Saliva was then collected at 15 minute intervals and its LDCL quenching propertied was tested. Note: That even after 120 minutes saliva still had enhanced antioxidative properties, suggesting that coffee derived polyphenols were avidly suck to oral surfaces and persisted there despite a constant salivary flow. (n = 3).

A similar long-retention of Folin-positive agents in saliva was also observed either after chewing dark chocolate **(** **Figure 10**) or after holding in the mouth, a cinnamon extract **(** **Figure 11** **).** Similar results were also obtained either with green tea, a pomegranate and cherry drinks (not shown) as well as with black tea (see [30]).

The article "The Oxidant-Scavenging Abilities in the Oral Cavity May Be Regulated by a Collaboration among Antioxidants in Saliva, Microorganisms, Blood Cells and Polyphenols: A Chemiluminescence-Based Study" was published in 2013. Journal: PLoS One.

**Figure 10:** A prolonged retention in the oral cavity of antioxidants from 10 gr of dark chocolate after chewing for 30 seconds as measured by LDCL. Note that even after 90 minutes saliva still has enhanced LDCL-quenching abilities indicating the high avidity of chocolate-derived polyphenols to oral surfaces. (n = 4).

**Figure 11:** The use of the Folin reagent to quantify cinnamon polyphenols in the oral cavity. Cinnamon powder was suspended in boiling water and the supernatant fluid containing 35 mM of polyphenols (GAE) was held in the mouth for 30 seconds and then eliminated. Note that even after 300 minutes Folin-positive agents were still retained in elevated amounts in the flowing saliva, indicating the high avidity of cinnamon polyphenols to oral structures and surfaces. (n = 3).

The results presented in **Figures 9** **,** **10** **,** **11** stress that “sticky” polyphenols may maintain a higher antioxidant status in the oral cavity, which might counteract the harmful effects of excessive ROS.

### Saliva Acts in Concert with Platelets, *Candida albicans* and with Polyphenols to Increase OSA

In previous studies, we employed catalase-positive RBC as sources of antioxidants. Since platelets extravasated from injured capillaries together with RBC are also extremely rich in catalase and since platelets play a major role in primary hemostasis, it was also of interest to establish whether similarly to RBC, platelets might also engage in a cross talk with salivary antioxidants, microbial antioxidants and polyphenols to increase OSA. We first prepared complexes between platelets (5×108) and quercetin (200 µM) and C. albicans (108/mL) and quercetin, washed them to remove unbound polyphenols and then interacted the complexes with saliva.

**Figure 12** shows that while both catalase-positive Candida and catalase-positive platelets induced typical bell-shaped patterns of light quenching, saliva at 20 µL had only a marginal OSA effect. On the other hand, combinations either between saliva and platelets, platelets-quercetin complexes, quercetin or platelets and quercetin, induced a marked OSA. However, a marked decrease in OSA occurred when either the catalase-rich platelets or Candida cells, had been pre-incubated for 30 seconds with 1 mM of sodium azide, to inactivate heme-proteins (not shown). It was also found (not shown) that the same patterns of fluorescence inhibition occurred with a variety of additional polyphenols, and fruit beverages.

The article "The Oxidant-Scavenging Abilities in the Oral Cavity May Be Regulated by a Collaboration among Antioxidants in Saliva, Microorganisms, Blood Cells and Polyphenols: A Chemiluminescence-Based Study" was published in 2013. Journal: PLoS One.

**Figure 12:** LDCL quenching patterns resulting from combinations among washed catalase-positive *Candida albicans* (CAND, 108/mL), saliva (20 µL), platelets (PLTs, 109/mL) and quercetin (5 µM) complexes were first prepared between platelets (PLTS) and quercetin and candida and quercetin. These were then interacted with saliva. Note that while compared to cocktail saliva alone had no OSA effect, candida induced a typical bell-shaped pattern of luminescence quenching. Combinations among the agents induced a progressive synergistic inhibition of light quenching. Similar results were also obtained if platelets were replaced by washed RBC (not shown).(n = 5).

## Discussion

The results presented propose a novel approach to evaluate how the antioxidant - oxidant balances in the oral cavity might be manipulated due to multiple interactions expected to occur on a daily basis among salivary antioxidants, microorganisms, blood elements and polyphenols from nutrients. The use of a highly sensitive luminol-dependent chemiluminescence assay to evaluate OSA resulting from multi-component systems is simple to perform, highly reproducible and also allows rapid quantifications of the OSA of whole bacteria, mammalian cells and cells coated by poly phenols.

Our study claims that:

1. The antioxidant status in the oral cavity, considered a “bio-reactor” [26], [31], might be under a constant balance due to synergistic interactions among the antioxidants of saliva, the oral microbial flora, polyphenols from nutrients and blood elements extravasated from injured capillaries.
2. Antioxidants may counteract the toxic oxidants generated on a daily basis in the oral cavity. These include peroxide, thiocyanous acid, and oxidants generated by activated neutrophils, which accumulate in infectious sites.
3. While most of the OSA activities of whole saliva are located in the supernatant fluids, saliva lost most of its OSA upon dialysis in tubings with a cutoff point of 6 kD, (**Figure 6**) indicating that the main antioxidant of saliva are associated as already suggested with low molecular-weight agents mainly, uric acid, ascorbate, reduced glutathione and albumin [1], [7]–[10].
4. Either whole saliva, salivary high molecular-weight agents retained after dialysis (**Figure 6** **),** mucin (**Figure 5**), human serum albumin or plasma, and also small amounts of ethanol (**Figure 3**), could all increase the “solubility” and availability of allegedly water-soluble antioxidant polyphenols, present in aqueous fruit beverages (**Figures 3** **,** **4** and also [16].
5. Saliva markedly enhanced OSA of complexes formed among RBC, platelets, bacteria and polyphenols (**Figures 7** **,** **8** **and** **12**).
6. Polyphenols from beverages which avidly bind to oral surfaces are retained there for long periods despite a constant salivary flow (**Figures 9** **,** **10** **,** **11**).
7. The OSA of saliva is probably the sum result of LMWA, polyphenols from nutrients, blood elements and mainly catalase-positive microbiota. Combinations among the 4 agents may bestow upon the oral cavity a substantial enhanced redox properties leading to a more efficient protection against oxidative stresses. Such possible interactions are demonstrated in a proposed scheme (**Figure 13**).

The article "The Oxidant-Scavenging Abilities in the Oral Cavity May Be Regulated by a Collaboration among Antioxidants in Saliva, Microorganisms, Blood Cells and Polyphenols: A Chemiluminescence-Based Study" was published in 2013. Journal: PLoS One.

**Figure 13:** Multiple collaborations among salivary and oral microbiota oxidants-antioxidants, blood elements and polyphenols from nutrients solubilized by mucin and albumin. These may regulate the redox status in the oral cavity and help to secure its integrity in health and in disease states.

In our study we first demonstrated that whole un-stimulated saliva possesses a capacity to decompose both ROS and RNS (**Figures 1a and 1b** **).** However, the luminescence quenching patterns, which measured oxidant scavenging, differed in the tow cocktails used. While H_2_O_2_ cocktail measures a flux of light, generated by preformed peroxide and OH. [23], the SIN-1 assay measures the alterations in the generation of the end product, peroxynitrite, resulting from the interaction of superoxide and NO. [3].

The OSA of saliva is mainly contributed by LMWA antioxidants [7]–[10], [32] localized in supernatant fluids, and was lost to a very large extent following dialysis in tubing with a cutoff point of 6 kD. However, as measured by luminescence, the ID 50 levels of fasting saliva in normal donors which ranges from 20–30 µL **(** **Figure 1a and b** **)** may be altered either by polyphenols from nutrients or also by small amounts of fresh blood extravastaed from injured capillaries. This may occur either following tooth brushing, use of tooth picks, during orthodontic treatments and in inflammatory sites. The ability of small amounts of ethanol to markedly increase OSA of saliva (**Figure 3**) indicates that poorly-soluble lipophilic antioxidant agents in red wine can be better solubilized and made more available as effective antioxidants due to its ethanol content**.** This phenomenon may therefore, shed more light on the role of ethanol in red wines, rich in polyphenols, as agents capable of neutralizing advanced lipid peroxidation end products generated in the stomach following consumption of fatty meats [26]. This also suggests that swallowed saliva rich in mucin (**Figure 5**), an agent which coats the oral cavity and also the stomach (see below), can combine with ethanol, rendering not only red wine polyphenols, but also many fruit beverages rich in polyphenols, more “soluble“ and thus able to better scavenge harmful oxidant species [16]. We also suggest that salivary albumin considered a “universal carrier” of metabolites and capable of forming complexes with polyphenols [27], may also contribute to a more efficient solubilization of lipophilic polyphenols.

The article "The Oxidant-Scavenging Abilities in the Oral Cavity May Be Regulated by a Collaboration among Antioxidants in Saliva, Microorganisms, Blood Cells and Polyphenols: A Chemiluminescence-Based Study" was published in 2013. Journal: PLoS One.

The role of high molecular weight salivary proteins as solubilizers of polyphenols (**Figures 4** **,** **5** **,** **6**) may also be important since it may explain the beneficial effects of polyphenols as potential attenuators of oxidative stresses related to cardiovascular events seen in populations which consume red wine together with fatty meats, the famous “French paradox“ [26], [33].

However, since the activity of mucin and albumin could be replaced by fresh heparinized plasma and also by cows’ and soy milk (not shown), it indicates the central role played by proteins as “solubilizers” of lipophilic antioxidant polyphenols and their potential nutritional importance.

Since RBCs as well as platelets are always regularly found in the oral cavity, in variable amounts, the findings that a marked enhancement of OSA can be induced by mixing saliva either with RBC (**Figure 7** **)** or with complexes formed between RBC and a polyphenols **(** **Figure 8**) are important observations. These suggest why even very moderate amounts of blood in the oral cavity may contribute to an enhanced redox status. The same rational can be applied for platelets as a potential source of antioxidant effect in the oral cavity as well (Figure 12).

The capacity of “sticky polyphenols” to adhere to RBC [13]–[16] also led to examine how long after holding in the mouth for short periods fruit beverages rich in polyphenols, saliva may still contain enhanced amounts of polyphenols presumably due to their ability to avidly bind to oral surfaces. This was tested by luminescence and also by the employing the Folin reagent which measures hydroxyl groups in polyphenols. **Figures 9** **,** **10** **,** **11** demonstrate that enhanced levels of Folin-positive agents are detected in saliva hours after the consumption of beverages. This implies that binding polyphenols to oral surfaces may function as a slow release devise capable of maintaining enhanced OSA. The ability of tea polyphenols to persist in the oral cavity was also previously reported by Lee et al. [30].

However, one cannot ignore the possibility that polyphenols, mainly tannins, the main causes of astringency**,** can rapidly bind to salivary proline-rich proteins, which undergo precipitation [34], [35] which facilitates their fast removal by salivary flow. However, since the amounts of polyphenols consumed by beverages are often in the millimolar levels, the loss of polyphenols by binding to proline-rich proteins might be negligible.

The article "The Oxidant-Scavenging Abilities in the Oral Cavity May Be Regulated by a Collaboration among Antioxidants in Saliva, Microorganisms, Blood Cells and Polyphenols: A Chemiluminescence-Based Study" was published in 2013. Journal: PLoS One.

The oral cavity is highly rich in microbiota, which possess both intracellular and surface-associated antioxidant agents. We therefore may also postulate that colonizing, opportunistic catalase-positive microbial species, might act in concert with the antioxidants of saliva, platelets, RBC, plasma and polyphenols from nutrients to create a higher antioxidant environmental status. Such multiple interactions leading to the collaborated enhanced scavenging of ROS is shown in **Figure 12** **,** where suspensions of catalase-rich *Candida albicans* and complexes formed between Candida cells and the polyphenols quercetin, acted in concert with catalase-rich platelets and with saliva to scavenge enhanced amounts of ROS. Similar results were also obtained using the cataslase-positive *Staph. Aureus* and *E. Coli* (not shown).

This experimental model indicates that the total OSA of the oral cavity is due to a sum effect of the antioxidant activities of saliva (LMWA, mucin and albumin), plasma antioxidants delivered via the crevicular fluid, the antioxidants associated with the microbial flora, blood elements and also “sticky” polyphenols [13]–[16], [30]. However, the balance between oxidants and antioxidants in the oral cavity might change drastically under pathological conditions. Therefore, a steady slow release of antioxidant polyphenols retained in the oral cavity, might be beneficial to cope with tissue damage. However, polyphenols from nutrients can also form redox couples with salivary ascorbate, where one antioxidant protects the other against oxidation (Ginsburg and Koren, un-published date) and also [36].

As summarized in **Figure 13**, collaboration among microbial oxidants/antioxidants and polyphenols from nutrients can create a complex redox balance which might directed towards two opposing directions, as pro- and antioxidants. This makes it difficult to evaluate the real redox status at any given time. Also, while a collaboration between microbial and host antioxidants might enhance resistance to oxidative stresses, excessive amounts of antioxidants might also compromise the protective role of neutrophils against microbial proliferations. Although polyphenols possess potent antioxidant and chelating properties, they might also act under certain conditions, also as pro-oxidants [37] and as signaling molecules [38], [39], capable of generating pro-inflammatory agonists. Furthermore, although the presence of blood in the oral cavity, might serve as “sinks” for ROS and as protectors of other cells against oxidative stress [12], iron released from hemolyzed RBC, might engage in the Fenton reaction to generate highly toxic hydroxyl radical [3]. One such an example is the long-term effects of experimental intra-cerebral hemorrhage caused by the release of iron from lysed RBC and leukocyte [40]. Therefore, enhanced antioxidant capacities in tissues might also act as “double-edged swords”. In addition to their antioxidant and metal chelating properties, polyphenols in beverages such as green tea, coffee, wine, cranberry and cinnamon drinks might also act as bactericidal agents [41] and also as inhibitors of the attachment of microorganisms to cell surfaces [42], [43]. However, a slow and steady release of polyphenols from oral surfaces, their local interaction with salivary oxidants (peroxide, OH**.**, OONO-) and perhaps also down-stream in the stomach, also with hydroperoxide and aldehydes oxidants generated following consumption of fatty nutrients [26], might also contribute to prevent the access of toxic oxidant species to the blood circulation. There they might alter LDL and contribute to formation of foam cells. This further supports the assumption that the beneficial effect of polyphenols as oxidant scavengers is exerted mainly in the oral cavity and in the stomach [26], [43], [44].

The article "The Oxidant-Scavenging Abilities in the Oral Cavity May Be Regulated by a Collaboration among Antioxidants in Saliva, Microorganisms, Blood Cells and Polyphenols: A Chemiluminescence-Based Study" was published in 2013. Journal: PLoS One.

Taken together, oxidative stresses anywhere in the organism can result from an imbalance of pro-oxidants and antioxidants involving excessive destructive free radical chemistry (See ref. [1], [33], [44], [45] and **Figure 13**), necessitates further studies in order to shed more light on the pros and cons of creating balanced oxidant-antioxidant status in the oral cavity and its possible role in oral pathologies. Saliva is therefore an ideal milieu to study non-invasive complex host-parasite interrelationships where the balances between oxidants and antioxidants play an important role in the integrity of oral tissues. However, since both microorganisms and host cells share potent catalase activities, it is paradoxical perhaps that microbes and the host may collaborate in an adverse manner to alter the complex redox status in the oral cavity.

Finally, one friendly advice to all food consumers: chew your food well, allow saliva to increase the solubilization of plant and fruit polyphenols making them more effective antioxidants [17]. This will introduce into the stomach effective antioxidants capable of neutralizing malondialdehydes (MDA) and hydroperoxides generated by fatty foods which, if not neutralized *in situ,* will eventually reach plasma to oxidize LDL [26], [46]. Therefore, always try consuming fatty foods simultaneously with polyphenols-rich fruit beverages.

The article "The Oxidant-Scavenging Abilities in the Oral Cavity May Be Regulated by a Collaboration among Antioxidants in Saliva, Microorganisms, Blood Cells and Polyphenols: A Chemiluminescence-Based Study" was published in 2013. Journal: PLoS One.

Lastly, the use in this study of a luminescence assay to quantify OSA proved highly reliable, reproducible and easy to perform, which allows quantifying the major intracellular antioxidants in red blood cells, platelets, catalase-positive microbiota and also antioxidant agents attached to surfaces of microbial and host cells. The combined use of luminescence and the determinations of polyphenols attached to cells by the Folin method is highly recommended as means to evaluate collaboration among antioxidants in saliva, bacteria, polyphenols and blood elements.
